# The Combination of Tradition and Future: Data-Driven Natural-Product-Based Treatments for Parkinson's Disease

**DOI:** 10.1155/2021/9990020

**Published:** 2021-07-14

**Authors:** Zhijun Miao, Jinwei Bai, Li Shen, Rajeev K. Singla

**Affiliations:** ^1^Institutes for Systems Genetics, Frontiers Science Center for Disease-related Molecular Network, West China Hospital, Sichuan University, Chengdu 610041, Sichuan, China; ^2^Department of Urology, Suzhou Dushu Lake Hospital, Suzhou, China; ^3^Library of West-China Hospital, Sichuan University, Chengdu 610041, China; ^4^iGlobal Research and Publishing Foundation, New Delhi 110059, India

## Abstract

Parkinson's disease (PD) is a neurodegenerative disorder in elderly people. The personalized diagnosis and treatment remain challenges all over the world. In recent years, natural products are becoming potential therapies for many complex diseases due to their stability and low drug resistance. With the development of informatics technologies, data-driven natural product discovery and healthcare is becoming reality. For PD, however, the relevant research and tools for natural products are quite limited. Here in this review, we summarize current available databases, tools, and models for general natural product discovery and synthesis. These useful resources could be used and integrated for future PD-specific natural product investigations. At the same time, the challenges and opportunities for future natural-product-based PD care will also be discussed.

## 1. Introduction

Parkinson's disease (PD) is a neurodegenerative disorder (NDD) commonly seen in the elderly. The prevalence of PD is increasing with age, of which the lifespan risk is 2% for men and 1.3% for women [1]. Many factors have been revealed to tightly relate to PD, including genes, gut microbes, the living environment, and lifestyle [2–4]. In the past decades, efforts have been made both in mechanism investigations and clinical treatments. A large number of molecules have been reported for their therapeutic potential against Parkinson's disease, such as levodopa [5], ubiquinone [6], and creatine [7]. The efficacy, however, is rather limited along with uncontrolled side effects [8]. Since several years ago, natural products have drawn more and more attention, which are considered as potential breakthroughs for PD treatments.

Natural products are a class of chemical compounds or substances produced by living organisms, the sources of which can be plants, animals, fungi, and bacteria [9]. Compared to synthetic drugs, natural products tend to have unique structures that are rather difficult to be synthesized in the lab. Nevertheless, the stabilities and efficacies sometimes are better [10]. Meanwhile, components in natural products are usually in the form of a mixture. Interactions among them result in weaker toxicity, side effects, and drug resistance [11,12]. Considering these advantages, an increasing number of research has been focusing on improving PD treatments with natural products. In a recent study, for example, gardenin A has shown its role in neuroprotection against environmental-toxin-induced Parkinson's disease pathogenesis [13]. Another study by Haruka et al. pointed out that sesaminol may increase Nrf2 expression and then activate the Nrf2-ARE signaling pathway and decrease the expression level of *α*-synuclein, indicating its preventative effect on PD [14]. Besides, Liu et al. also found that a fumarate salt form of dimethylaminomicheliolide called ACT001 derived from parthenolide can prevent the overexpression of *α*-synuclein induced by 1-methyl-4-phenyl-1, 2, 3, 6-tetrahydropyridine, which could serve as a good concomitant drug for L-3, 4-dihydroxyphenylalanine (L-DOPA) to lower the intake dose and its side effects [15]. These gathering evidence show a great therapeutic potential of natural products in PD treatments.

Traditional drug discovery is mainly based on two approaches: ligand-based drug design and structure-based drug design [16]. Computational technologies are frequently applied during this period, which is usually known as Computer-Aided Drug Discovery (CADD). Over the past decades, the innovations in chemistry, biomedical science, and engineering, as well as high-throughput screening, have rapidly improved the efficiency of a huge number of compounds' screening for 1–3 specific targets. Numerous tools, databases, and models are constructed with accumulating data [17], bringing current drug discovery into the “big data era.” There are five intrinsic characteristics for big data, including volume, variety, value, velocity, and veracity [18], as shown in Figure 1. Compared to traditional CADD methods, a successful big-data-based CADD strategy firstly needs a standard for integration of multilevel data. At the same time, high-speed algorithms are required for data mining, structuring, and analysis in order to ensure the efficiency and accuracy for drug-target interaction simulation. Finally, the main roles for most previous databases are storage and reference. The density of data value is pretty low. How to utilize updated technologies and algorithms to figure out the real value of data will be very essential for novel drug discovery. In summary, it is necessary to develop novel approaches that systematically address the high-volume, multidimensional, and highly sparse data sources needed for drug efficacy and adverse effect prediction and evaluation.

In recent years, some studies have already employed computational methods on natural product identification and characterization. These resources could be quite valuable for PD-related natural product discovery. In this review, we will summarize available data sources, databases, computational tools, and models and, last but not the least, the future challenges and chances for data-driven natural product discovery for PD treatments.

## 2. Natural Product Databases for Data Sharing and References

Biomedical studies have made great advances with the development of omics and informatics technologies. Accumulating scientific data, including omics data, clinical data, and other biological data, are extremely valuable research resources. Thus, data standardization, annotation, sharing, and integration are becoming quite essential. The well-structured databases can not only store and manage existing data but also can be utilized for data sharing and integrated analysis. Good examples for such databases in PD research include NDDVD [19], Gene4PD [20], and PDmethDB [21]. Natural products have a broad range of compounds, and a large number of diseases can be treated by them. The establishment of relevant databases can greatly facilitate our understanding towards the mechanisms by which a certain natural product works on its target diseases, and clinicians can also get advised for precision treatments [22]. To date, there are already quite a few published natural-product-specific databases. Although Sorokina et al. have constructed a database named COCONUT (https://coconut.naturalproducts.net) where they collected a part of free available databases for natural products [23], we will make up and summarize some nonincluded databases for reference, the list of which is shown in Table 1.

### 2.1. Databases of Different Traditional Medicine Systems

Traditional medicine can be divided into several medical systems according to the regions, such as traditional Chinese medicine (TCM), traditional Indian medicine (also known as Ayurveda), and traditional Islamic medicine. Although there are overlaps between different traditional medical systems, they also have their own unique features. From a systemic view, databases and knowledge bases to share and annotate these medical systems is the first step for integrated analysis and natural products screening. Efforts have been made in the past decades. For example, Fang et al. built a comprehensive database for traditional Chinese medicine called HERB, in which the basic herb information, effective targets, and gene-gene interactions are provided [24]. Another TCM-related database is SymMap, which could be a good support for HERB as it contains not only prescriptions but also symptom mappings for users [32]. The Indian Medical Plants, Phytochemistry And Therapeutics (IMPPAT) is a curated database for Indian traditional medicine that shares the standardized names and usages of some traditional Indian herbs [33], and for Irian traditional medicine, there is also a similar database called Universal Natural Product Resource (UNaProd) [29]. A direct evidence among these databases is Atropa acuminata, which was reported to be a potential natural product medicine for PD. The effective compound named atropine is demonstrated to remarkably reduce raclopride-induced muscle rigidity through the activation of the ventral region of the striatum [39]. Meanwhile, there are also some indirect clues. For instance, isorhynchophylline, which is the compound of *Uncaria sessilifructus, Uncaria tomentosa,* and *Semen Cavaliae*, can significantly promote autophagy of neuronal cells and avoid the accumulation of *α*-synuclein by targeting SCNA [40]. Curcumin derived from *Acorus calamus* and *Radix Angelicae sinensis* can notably inhibit the activity of LRRK2 kinase and suppress PD-like phenotypes [41]. Taken together, these databases are mainly from a clinical view, data from which may provide us with potential traditional medicine prescripts for PD treatments. At the same time, integrated analysis of them may give novel insights to researchers and clinicians from different regions. Real-time update, thus, is quite essential.

### 2.2. Databases of Different Natural Product Sources

Natural products have multiple sources. An unfractionated extract from these sources may contain a range of structurally diverse and often novel chemical compounds [42]. The biological diversity contributes to the chemical diversity in the nature; in other words, researchers have to collect samples all over the world for natural product screening and novel drug discovery [43]. During this period, databases for such data collection are highly demanded. There are two main roles for these databases. First, they are data containers. Second, they can serve as references. Once potential natural products are identified, a comparison could be conducted with known products in the databases between their compounds, structures, and so on [44]. Also, advanced molecular-level analysis can be performed for further mechanism investigation and target screening. In the past decades, several such databases have been already constructed, including NPASS [44], NANPDB [45], and Super Natural II [46], most of which were included or introduced in COCONUT. Recently, there are several newly published resources which are good supplementary for natural product source databases. For example, Xu et al. built a relationship database called Natural Products & Biological Sources (NPBS), which is an online resource that contains relationships between natural products and biological sources [26]. Compared to previous natural product databases, NPBS not only provides molecular properties and biological sources of natural products but also shows properties of biological sources. There are some other databases which focus on specific classes of natural products. For instance, the Comprehensive Marine Natural Products Database (CMNPD) is a database for marine-sourced natural products, whereas the *Pseudomonas aeruginosa* Metabolome Database (PAMDB) is a resource for *Pseudomonas aeruginosa* metabolome [28,34]. Network analysis and ontology analysis are inserted. These databases could serve as good references when we do novel natural product screenings for PD treatments.

## 3. Computational Models and Tools for PD Natural Product Investigation

Computational modeling is a powerful method for PD diagnosis, treatments, and drug discovery. Statistical tests, such as *t*-test, Wilcoxon signed-rank test, and eBayes, are commonly used for dysfunctional molecule identification [47]. Combined with network-based analysis, these significantly dysfunctional molecules can be further investigated for their potential as biomarkers or therapeutic targets for PD [22]. In recent years, with the assistance of deep learning, the drug target screening has entered into a new era. AlphaFold, for example, is a deep-learning-based prediction tool for protein folding, which remarkably increased the target discovery efficiency [48]. How to integrate and utilize these resources well will be the key for future natural product investigation and PD care [49].

### 3.1. Models for Natural Product Synthesis

The production of natural products via extraction from biological organisms is often limited several factors, including slow growth, low yield, extraction and purification efficiencies, and weather and climate change. Laborious synthesis could be a quite accessible way for high-volume natural product production. However, it is always a challenge for computer-aided organic synthesis. Although there are already some tools and algorithms which are capable of completely autonomous planning, these programs can only execute one step at a time. In most cases, the computer-aided drug design and target screening are limited to relatively simple targets. Chematica, which was designed by Mikulak-Klucznik et al., is a tool for complex natural product syntheses route design [50]. With the input of reactants, steps, and target products, a highly efficient synthesis route can be designed in seconds. Compared to the reported synthesis routes, the steps taken in newly designed routes are less and the efficiency is higher, and the cost is lower as well [51]. Another route design tool developed by Waller et al. is in a different way [52]. Monte Carlo tree search was applied in this system for retrosynthetic route discovery, as shown in Figure 2. With the assistance of symbolic artificial intelligence, this new AI tool does not require chemists to input any rules, but learns the rules of chemical transformation on its own and then performs fast and efficient inverse synthesis analyses based on reported one-step reactions. When asked to design a synthetic route for a target molecule, this AI system can make selections and judgements by itself and select the most promising precursor molecule based on the design rules. Feasibility of the synthesis will be further evaluated until a best route is found. This is a sensational innovation as it can create new strategies to find the best way for target molecule syntheses, totally without relying on any existing experience or strategies. Taken together, these tools discussed above could serve as strong tools for natural product laborious synthesis design.

### 3.2. Models for Precise Natural Product Medication

Network is an important physics theory which has been applied into many fields [53]. The application of that in biomedicine enables us to measure different molecule interactions at the systemic level [54]. Previous biomedical studies tended to utilize biological networks to investigate the consequences to the whole systems brought by dysfunctional molecules [55]. A more functional application is to use protein-protein interaction, gene-gene interaction, or coexpression network for complex disease biomarker discovery and drug target screening [56–59]. In the “Genomic Era,” DNA/RNA sequencing has enabled rapid identification of new targets and reuse of approved drugs to treat heterogeneous diseases by “precise” targeting of personalized disease modules [60]. The network-based approach makes it possible for drug retargeting and combination therapy by measuring the proximity of disease proteins in the human protein interaction group. Cheng et al. developed a genome-wide position system named Genome-wide Positioning Systems network (GPSnet), which can reuse drugs via specific disease module targets derived from an individual patient's DNA and RNA sequencing profiles mapped to the human protein-protein interactome network [61]. Two main functions are included in GPSnet: cancer specific disease module identification and computational drug repurposing. Random walk with restart process was applied for cancer-specific disease model identification, after which network distance between node *s* and nearest disease protein *t* was measured through the following formula:

(1) $$\begin{array}{c} d\left(S,\;T\right)\;=\;\frac{1}{\left\|T\right\|}\underset{t\in T}{\sum }\min_{s\in S}d\left(s,\;t\right). \end{array}$$

Here, S is the set of disease proteins, and *T* is the set of drug targets. The significance of the network distance between a drug and a given disease was further evaluated by setting a reference distance distribution. GPSnet may be a promising tool for natural product discovery, synthesis, and precise usage in PD treatments. Besides, there are also studies which applied network theory for natural products' potential in human health. Cao et al. employed a metabolome- and metagenome-wide association network to distinguish microbial natural products and microbial biotransformation products in human microbiota [62]. Chamberlin et al. analyzed a natural product-target interaction network and claimed that natural products show target family groupings both distinct from and in common with cancer drugs, showing tremendous potential of natural products in cancer therapy [63]. Another study by Gogoi et al. also provides similar evidence via pharmacology network analysis [64]. Although there are still no studies which applied network analysis to PD-specific natural product investigation, with the help of could computing and the evidence above, there could be great chances in the future.

## 4. Perspectives on Big-Data-Based PD Natural Product Medicine

In the big data era, PD care barely depends on clinical treatments. The involvement of informatics technologies has tightly combined basic research and advanced technologies in hardware development and clinical medicine, together promoting PD care into the “precision medical care era” [65]. In the last decade, technologies such as virtual reality and augmented reality, robot, and wearable devices have developed numerous strategies for PD prevention, diagnosis, and treatment [66], which has become an indispensable part for big-data-based PD medicine.  Figure 3 shows a blueprint for future informatics-assisted PD care. First, huge databases for multilevel data storage, including omics data, clinical data, lifestyle data, environment data, and natural product data, are demanded. These data resources may provide references and knowledge for AI training. A well-trained AI system based on them will then play 2 main roles. On one hand, the system can be utilized for novel natural product screening and precise drug recommendation, which is slightly similar to GPSnet. On the other hand, with real-time physiological data as references, the system can monitor patients' health status and work as an alarming system. Meanwhile, daily analysis on the cloud platform can also provide PD care suggestions for PD patients. To realize such health care scheme, however, there are still several challenges need to be solved.

### 4.1. Databases and Knowledge Bases for PD-Specific Natural Products

Current natural product databases only stored very limited candidates for PD treatments. As the relevant research data accumulate, however, a PD-specific natural product database is urgently needed for future therapeutic compound screening. Since PD is a complex disease, a systematic analysis should be integrated into the database as well. As data are gathered from a different level, such as effective compounds in natural products, supportive molecules, targets, environments, and other PD-associated factors, a knowledge base could be further constructed, which will draw a multilayered landscape for PD care. Based on the constructed knowledge bases, a knowledge graph, which is a resource that integrates one or more expert-derived sources of information into a graph where nodes represent biomedical entities and edges represent relationships between two entities, will be a good support, giving novel and clear insights for both clinical decision and basic research [67].

### 4.2. AI-Based Systematic Modeling for Highly Efficient Natural Product Screening

Since PD is the product of a dynamic interaction between the patient's genetics, modeling for the evolution of PD and dynamic simulation of the effects of natural products on PD patients is the key for the AI system. To identify the key factors for PD development and figure out highly efficient natural products will be a challenge [68]. Meanwhile, as data accumulate, how to improve the accuracy and efficiency of AI systems for natural product screening and precise medication is another challenge. Under this situation, training data quality, feature extraction, algorithm selection and optimization, and validation are the most important parts for improvements. A standard for data collection and data clear is essential as well.

### 4.3. Integration of Cross-Level Data to Assist Precision PD Treatments

PD research and medication covers a broad range of data types, which are from molecular phenotypes to clinical phenotypes. The connections between them tend to be quite complex. At present, studies usually focus on only few parts and the data generated are isolated. The linkage between molecular phenotype and clinical phenotype are important for disease systemic modeling. An example is that a certain natural product is utilized and positive changes are noticed in the molecular level but nothing happened on patients' clinical phenotypes. Thus, if molecular-clinical paired data are collected over time, the progression of PD can be, therefore, simulated and modeled. There are already several mature paradigms such as The *Cancer* Genome Atlas (TCGA) and International *Cancer* Genome Consortium (ICGC), which could be excellent references for PD data integration.

## Figures and Tables

**Figure 1:** “5V” characteristics of big data.

**Figure 2:** The Monte Carlo tree search algorithm for synthesis route design.

**Figure 3:** A systemic structure of data-driven PD care.

**Table 1:** A summary on natural product databases which are not included in COCONUT.

Name	Description	Url	Pmid	References
HERB	A traditional Chinese medicine database providing basic herb information, effective targets, expression profiling, and interaction networks	https://herb.ac.cn	33264402	[24]
PSC-db	A 3D database for plant secondary compounds	https://pscdb.appsbio.utalca.cl	33672700	[25]
NPBS	A database containing relationships between natural products and biological sources	https://www.organchem.csdb.cn/scdb/NPBS	33306802	[26]
BiG-FAM	A biosynthetic gene cluster families database	https://bigfam.bioinformatics.nl	33010170	[27]
CMNPD	A database of marine natural products	https://www.cmnpd.org	32986829	[28]
UNaProd	A natural products data resource for Iranian traditional medicine	https://jafarilab.com/unaprod	32454857	[29]
TeroKit	A database for terpenome academic research	https://terokit.qmclab.com	32286817	[30]
MedPServer	A database for therapeutic targets screening of natural products	https://bif.uohyd.ac.in/medserver	30381914	[31]
SymMap	A database for Chinese traditional medicine with symptom mapping	https://www.symmap.org	30380087	[32]
IMPPAT	An Indian medical plants, phytochemistry, and therapeutics database	https://cb.imsc.res.in/imppat	29531263	[33]
PAMDB	A database of *Pseudomonas aeruginosa* metabolome	https://pseudomonas.umaryland.edu	29106626	[34]
TriForC	A database for plant triterpene biosynthesis	https://bioinformatics.psb.ugent.be/triforc	29045755	[35]
DEREP-NP	A database for rapid dereplication of known natural products	https://github.com/clzani/DEREP-NP	28616931	[36]
TMDB	A database for small-molecule compounds from tea	https://pcsb.ahau.edu.cn:8080/TCDB/index.jsp	25224438	[37]
3DMET	A database for 3D structures of natural metabolites	https://www.3dmet.dna.affrc.go.jp	23293959	[38]

## Data Availability

The literature used to prepare this review article is already available publicly.
